The article "Anti-DDI Resource: A Dataset for Potential Negative Reported Interaction Combinations to Improve Medical Research and Decision-Making" was retracted in 2023. Reasons: unreliable results or conclusions; concerns about the data; concerns about the peer review; concerns about the citations.

# Anti-DDI Resource: A Dataset for Potential Negative Reported Interaction Combinations to Improve Medical Research and Decision-Making

**DOI:** 10.1155/2022/8904342

**Published:** 2022-04-09

**Authors:** Abdullah Assiri, Adeeb Noor

**Affiliations:** ^1^Department of Clinical Pharmacy, College of Pharmacy, King Khalid University, Abha 62529, Saudi Arabia; ^2^Information Technology Department, Faculty of Computing and Information Technology, King Abdulaziz University, Jeddah 21589, Saudi Arabia

## Abstract

Potential drug-drug interactions (DDIs) are a core concern across medical decision support systems. Among healthcare practitioners, the common practice for screening these interactions is via computer software. However, as real-world negative reporting is missing, counterexamples that serve as contradictory evidence may exist. In this study, we have developed an anti-DDI resource, a set of drug combinations having negative reported interactions. This resource was created from a set of the top 200 most-used drugs, resulting in 14365 prospective negative reported DDI pairs. During analysis and filtering, 2110 DDIs (14.69%) were found in publicly free DDI resources, another 11130 (77.48%) were filtered by a rule-based inference engine incorporating ten mechanisms of interaction, and 208 were identified through commercial resources. Additionally, 90 pairs were removed due to recent FDA approvals or being unapplicable in clinical use. The final set of 827 drug pairs represents combinations potentially having negative reported interactions. The anti-DDI resource is intended to provide a distinctly different direction from the state of the art and establish a ground focus more centered on the evaluation and utilization of existing knowledge for performing thorough assessments. Our negative reported DDIs resource shall provide healthcare practitioners with a level of certainty on DDIs that is worth investigating.

## 1. Introduction

In the course of primary care, patients often are prescribed drugs that might have a risk of interaction, and the majority of such interactions are of major relevance [1]. Adverse interaction of drugs may lead to hospital admission and serves to increase morbidity and mortality. Additionally, several studies have reported an increase in patient hospital stay when DDIs are identified, suggesting that DDIs have a significant clinical and economic burden. Accordingly, ensuring quality pharmacotherapy requires the selection of appropriate drug combinations considering the condition being treated [2]. As concerns patient factors, this means considering cost, dosage, administration method, contraindications, and possible adverse reactions; but the prospect of one drug impacting another in terms of its safety or efficacy—that is, a drug-drug interaction (DDI)—is also not to be ignored [2, 3].

Conceptually, it is common practice to screen potential interactions via computer software, and numerous programs developed for identifying drug interactions presently see wide use in detecting interactions of clinical significance. For example, the commercial resources Lexicomp [4] and Micromedex [5] have been utilized by healthcare practitioners in detecting and determining the risk of interactions. Other publicly available free resources, such as DrugBank [6] and Drugs.com [7], are also widely leveraged for reporting known and potential interactions. However, despite the importance of DDI detection, existing DDI resources have a low level of overlap and a high level of diversity in reported interactions. For example, a recent study conducted by our group [8] demonstrated considerable variation among five commercial and free resources when used in reporting chemotherapy agent interactions.

As a result, it is common that available resources, whether commercial or publicly free, fail to detect all significant interactions, yield alerts whose significance is questionable, and do not supply information on risk factors for adverse reactions [9–11]. One reason for the diversity in these resources is that each software has been developed to employ a different algorithm and database combination [12–14]. Another is that the determination of related literature primarily depends on expert evaluation, ultimately leading to discrepancies in the references that different utilities incorporate. A third is the lack of a robust validation process for algorithms [9]. Consequently, this problem may be alleviated, at least in part, by instituting precise, clear instructions for algorithm development and validation.

In fact, the lack of overlap among DDI resources seems to be more due to specialization of resources than to negative consideration (i.e., no reported interaction = potential safe interaction combination). While originally a larger number of utilities and resources were considered for input, the actual resources that ended up being used are those with clinical/research backing. Furthermore, investment in thoughtful research and clinical trials proves the worthiness of the reported DDIs. This does not consider information that was “omitted” for whatever reason (i.e., any found DDI is assumed to be reported). In healthcare practice, on the other hand, it is essential to be both selective and transparent when choosing drug interactions for inclusion in such resources. Nonetheless, among the abundance of available utilities, no particular resource has yet emerged as a groud-truth for healthcare practitioners.

Here, we present the development of a potentially negatively reported DDI dataset, the anti-DDI resource, containing the most commonly prescribed drug pairs for which no DDIs have been reported. This resource is created as a means of differentiation from the state of the art and to provide a different direction, establishing a ground focus centered more on evaluation than on the generation and utilization of expanded knowledge and resources to perform evaluations. To the best of our knowledge, this represents the first study to construct such a list by employing a data-driven approach in conjunction with widely-employed DDI-screening software, and with the output further reviewed by healthcare practitioners. This robustly-resourced, trustworthy dataset has the potential to benefit both healthcare practitioners and researchers in the course of their work; being comprised of the most frequently prescribed drugs, it serves to summarize common safe combinations along with those least utilized due to safety concerns. Finally, the anti-DDI resource can enable stratification of patients receiving multiple drugs according to risk for DDIs, and so benefit practitioners in reducing unwanted effects.

## 2. Materials and Methods

### 2.1. Data Baseline

All possible pairwise drug combinations were generated for a set of the top 200 drugs, which include those most commonly used to treat several conditions. The list of top drugs was obtained from [15]. The rationale was to develop the initial dataset from the most-used drugs, with which patients might be at higher risk of being exposed to DDIs. The list can vary slightly from year to year and country to country according to national health policies. When generating drug combinations, consideration was given to reasons other than DDIs that preclude drugs being used together, such as having similar indications or belonging to the same pharmacological group.

### 2.2. Drug List Curation and Drug Mapping

From the top 200 most-used drugs, we generated 14365 prospective negative reported DDI pairs. The steps of pair creation are detailed below:

(i) Step 1: we normalized each drug name in the list to the corresponding UMLS concept unique identifier (CUI) through UMLS terminology services (UTS) [16]. For each drug, we utilized the text search box provided by the UTS tool to extract the equivalent CUI. We also ensured that the retrieved CUI was grouped correctly in the UMLS semantic network, i.e. as a drug. This yielded 192 drugs, as there were eight drugs with no CUIs.
(ii) Step 2: we mapped the UMLS CUI of each drug to its STITCH ID using Anatomical Therapeutic Chemical (ATC) identifiers. This step was necessary to enable checking for interactions as reported and represented by the publicly free DDI resources. This step reduced the set to 170 recognized drugs.
(iii) Step 3: we created pairwise combinations of the 170 unique drugs as follows:
    For each drug in the list:
    Create a list of all possible pairs of drugs that could interact as a result of any combination.

This produced 14365 prospective negative reported DDI pairs.

### 2.3. Checking Prospective Negative Reported DDI Pairs against Publicly-Free DDI Resources

To ensure our final list consisted of only potential negative reported DDI pairs, we intended to remove any pair having been recorded in either clinical or computational DDI resources. Accordingly, we downloaded the potential drug-drug interaction (PDDI) knowledge base of Ayvaz et al. [17] from https://github.com/dbmi-pitt/public-PDDI-analysis, obtained on 01/02/2022. This database consisted of two files. The first, labeled “Conservative,” featured mappings based on both International Chemical Identifiers and either the drug preferred term or synonym. It contained the following DDI sources and corresponding potential DDI counts, for 200159 potential DDIs in total: Drugbank-24103, NDF-RT-1876, KEGG-52104, CredibleMeds-83, DDI Corpus 2011-334, DDI Corpus 2013-787, NLM Corpus-238, PK Corpus-146, ONC High-Priority-1930, ONC Non-Interuptive-2101, OSCAR-10325, HIV-19198, HEP-11194, FRENCH-62047, and World Vista-13693. The second file, labeled “Non-conservative,” featured mappings based just on International Chemical Identifiers or either the drug preferred term or synonym. It contained the following DDI sources and corresponding potential DDI counts, for 219617 potential DDIs in total: Drugbank-24103, NDF-RT-2606, KEGG-52104, CredibleMeds-83, DDI Corpus 2011-733, DDI Corpus 2013-1780, NLM Corpus-328, PK Corpus-184, ONC High-Priority-1930, ONC Non-Interuptive-2101, OSCAR-10325, HIV-19198, HEP-11194, FRENCH-62047, and World Vista-30901.

We integrated both sets and removed duplicate entries, which yielded a set of 40631 DDIs. After that, we tested our prospective negative reported DDI pairs as follows:

For each DDI in the possible negative set:

  Check for the interaction in all integrated DDI resources
  Retrieve all resources that report an interaction
  Remove the pair with the identified interaction
  Continue

This filtering reduced the list from 14365 to 12255, so 2110 of the prospective negative pairs were reported as interacting in the free resources.

### 2.4. Eliminating False-Positive Prospective Negative DDI Pairs Based on Mechanisms of Interaction

Following our construction of the list of prospective negative reported DDI pairs and testing it against publicly free DDI resources, we took the remaining 12255 pairs and annotated them with interaction mechanisms using the Drug-drug Interaction Discovery and Demystification (D3) inference framework by Noor et al. [14]. D3 applies rules on a knowledge graph to distinguish the following mechanisms of interaction: protein binding, metabolic induction & inhibition, transporter induction & inhibition, multiple pathways, competitive pharmacological, additive pharmacodynamic, indication similarity, and side-effect similarity. We removed any DDI from the prospective negative list that was identified as having a mechanistic interaction by the D3 system as follows:

For each DDI in the negative set:

  Apply D3 rules on the DDI pair
  If at least one rule is retrieved (a mechanism of interaction is found), remove the pair
  Else keep it

After this evaluation, the number of prospective negative pairs decreased to 1125. Therefore, more than 70% (11130) were found to be false positives, i.e. were explained by at least one mechanism of interaction included in the D3 framework.

### 2.5. Technical Validation by Experts and FDA Approval Cutoff for Quality Assurance of Prospective Negative Reported DDI Pairs

After generation and filtering of the set of pairwise combinations, two experts (trained, licensed pharmacists) reviewed the list for repetition and unapplicable drug combinations. Multiple criteria were established for the reviewers to follow. First, each pharmacist reviewed all generated combinations for repetitions in which the same two drugs were combined in different directions. Second, each pharmacist assessed the applicability of every drug pair to clinical practice and its clinical appropriateness or lack thereof. Lastly, agreement between the two pharmacists was assessed, with consensus being required for the removal of any pair from the dataset. Additionally, all drugs approved after 2018 were removed due to lacking sufficient reported DDI studies or DDI-associated adverse reactions.

### 2.6. Eliminating False Positives from Prospective Negative Reported DDI Pairs Based on Commercial DDI Resources

Finally, the list was checked for previously-reported potential DDIs by entering each pair into the well-known software Lexicomp [5]. The rationale for using Lexicomp over other resources was that it is considered a reliable resource for clinical information, and therefore is the most commonly used drug software among clinical and research institutions. DDI risk in Lexicomp is classified as follows: no known interaction (A), no action needed (B-minor), monitor therapy (C-moderate), consider therapy modification (D-major), and avoid combination (X-major). Drug pairs were considered as detected DDIs and removed from the dataset when classified in any class from B to X. Pairs labeled with class A were retained. All removed pairs were collected and reported as shown in Figures 1 & 2, after which a similar check was performed against Drugs.com [7]. DDI risk in Drugs.com is classified as follows: minor, moderate, or major interaction. Any pairs labeled with any of these classes were recorded and removed from the final dataset. Lastly, the final filtered list was reviewed by two trained and licensed pharmacists, in which process each pharmacist respectively reentered the drug pairs into one of the commercial DDI resources (either Lexicomp or Drugs.com) to confirm the absence of DDI risk among those included in the final list.

## 3. Data Records

The final list of potential negative reported DDI pairs evaluated in this study is publicly available as tab-delimited files upon request.  Table 1 gives a summary of the drug pairs, their validation, DDI risks, and risk stratifications, along with an outline of the available data files, which can be accessed directly through the corresponding URLs. Of the 14365 total drug pairs constructed from the set of 200 drugs, 827 (5.76%) were retained to comprise the final list, those having no potential risk for DDIs. In the course of the filtering process, 2110 DDIs (14.69%) were excluded based on available resources, and 11130 (77.48%) were identified by the D3 algorithm. Checking against Lexicomp and Drugs.com yielded 208 DDIs between them, of which 20 were reported in Lexicomp as requiring therapy modification, while 5 in Drugs.com were classed as major DDIs.

## 4. Limitations

The accuracy of this work is constrained by the data resources and by the computation methods. First, not all potential DDI mechanisms are incorporated into the D3 algorithm that was used for filtering potential DDIs, hence some DDIs might be missing. This limitation was moderated by checking the filtered list against two commonly-used resources, Lexicomp and Drugs.com. However, these resources have their own limits in being based on results from clinical studies that cannot be generalized to all populations. As such, the obtained list might be subjected to modifications as more clinical data become available. Our set of drug combinations represents a comprehensive list of pairwise combinations of the top 200 most-used drugs. In addition, validation of this dataset utilized all resources presently available; that said, future studies may produce new findings and new reports of DDIs that disqualify some of the “risk-free” combinations identified here. To help minimize this prospect, we only considered drugs that were approved before 2018 and so had enough data available to be confident in their safety. Furthermore, our study group will continue to annually update this list to ensure its ongoing accuracy.

## 5. Data Utility (Usage Notes)

### 5.1. Validation of DDI Prediction Software

As no negative reported DDI dataset is available for validation of DDI research, our group was inspired to develop a different means of validating newly-developed DDI prediction algorithms. Researchers can use this dataset, available upon request, alongside current validation methods to assess developed algorithms in terms of false-positive DDIs. Approaching validation from two directions will undoubtedly provide more precise and accurate assessments of prediction accuracy for new software.

### 5.2. Comprehensive List of Drug Combinations for Healthcare Practitioners

Given the discrepancies in reported DDIs among available public free and noncommercial resources, healthcare practitioners must have other means of detecting potential DDIs or confirming the safety of a given combination of drugs. Such capability enables the provision of appropriate patient care and the minimization of unwanted effects that stem from concurrent treatment with multiple drugs. Our dataset presented here represents an excellent first step towards a comprehensive list of drugs that can be safely utilized in combination, assuring the absence of DDI risk in patients. Additionally, it can guide healthcare practitioners by providing potential safe alternatives for interacting drugs. Notably, several drugs occurred with high frequency among drug pairs included in the final dataset, as shown in Table 1, indicating to some extent a degree of safe use for these drugs in clinical practice. Further extension of this work would have a significant impact in minimizing the frustrations that available DDI software poses for healthcare practitioners. In addition, a simplified version of this dataset can be made publicly available to patients as a reputable, trustworthy resource, reducing reliance on free resources of dubious validity that could mislead and provide imprecise information regarding drugs.

## 6. Discussion and Conclusions

In clinical pharmacy, understanding, and managing DDI events poses a major challenge. Several algorithms and strategies have been proposed by healthcare practitioners and researchers alike in attempts to address this perplexing subject. Our group previously developed a DDI prediction algorithm incorporating ten potential mechanisms [14, 18]; other algorithms have been developed to predict DDIs and stratify risk based on available DDI resources [19–21]. A persistent challenge in all of these endeavors is the lack of proper validation data for the developed algorithms [9].

This study extracted the top 200 most-used drugs from available resources and assessed all possible pairwise combinations of those drugs. Distinct from the state of the art, we filtered the generated list to identify those pairs having no risk of interaction. As no negative dataset of DDIs is yet available, we leveraged multiple resources for evidence of potential negative DDIs. In addition, the list was reviewed manually by experts to ensure the logic of generated combinations and the plausibility of their use in healthcare practice. The rigor of this filtering and review process ensures the resulting dataset is precise and well-constructed, and that it is appropriate for utilization in diverse situations.

As this approach of singling out safe drug combinations is unique in current DDI research, which predominantly focuses on the negative aspects of interactions and associated adverse events, it has the potential to open up new avenues and perspectives. Therefore, a wide range of researchers would significantly benefit from this work in many ways. Additionally, we plan to continue developing this work by integrating data from additional resources and considering all drugs with clinical use, not solely the most-used. We additionally plan to validate the clinical safety of all drug resources by connecting the generated combinations with data on their actual use.

In summary, the method employed here approaches research into DDIs and associated events from a new perspective and opens a new avenue for considering concurrently-used drugs on multiple levels. Further research is merited to address the challenges that yet limit DDI prediction algorithms and to improve clinical decision-making and patient safety in meaningful ways.

## Figures and Tables

**Figure 1:** Flowchart of dataset construction and validation processes.

**Figure 2:** Type distribution of DDIs identified through the dataset construction and validation processes.

**Table 1:** Description of anti-DDI resource.

Parameter	(*n*)	Comments
Total number of drugs	172	
Total number of drug combinations	827	
Technical validation	52	Duplication
Lexicomp	89	Known DDI
Drugs.com	119	Known DDI
Approved after 2018	38	Recent approval
Checker 1	0	
Checker 2	0	
Total	298	

*Detected DDIs*		
Minor	20	
Moderate	123	
Major	25	

*Medications most frequently appearing*		
Sevelamer	152	
Ustekinumab	140	
Levetiracetam	78	
Atenolol	77	
Liraglutide	72	

## Data Availability

The data generated by this work are available on supplementary 1.
